# Clinical Experience of Diagnosis and Surgical Treatment of 6 Cases of Acute Subhepatic Appendicitis

This article has been retracted.

**DOI:** 10.1155/2022/4969774

**Published:** 2022-04-16

**Authors:** Hongguo Yang, Junjie Jiang, Zhiming Hu, Bing Zhang, Wenwei Cai, Liming Xu, Kefeng Lu

**Affiliations:** ^1^Department of Hepatobiliary & Pancreatic Surgery, Tongde Hospital of Zhejiang Province, Hangzhou 310012, China; ^2^Zhejiang Chinese Medical University, Hangzhou 31001, China; ^3^Department of Emergency, Zhejiang Provincial People's Hospital, Hangzhou 310014, China; ^4^Department of Ultrasonography, Zhejiang Provincial People's Hospital, Hangzhou 310014, China

## Abstract

To summarize the experience of diagnosis and surgical treatment of 6 cases of acute subhepatic appendicitis. The clinical data of 6 patients with subacute appendicitis in Zhejiang Provincial People's Hospital from July 2018 to December 2019 were analyzed retrospectively. *Results*. There were 5 males and 1 female. All 6 cases were diagnosed as appendicitis by abdominal CT before operation. All patients underwent laparoscopic appendectomy without conversion to laparotomy. One case of ectopic appendix was located under the liver with absence of ascending colon, one case of ectopic appendix was located under the liver with ectopic ascending colon of transverse colon, one case of appendix head was located in the liver cyst, and the resection of liver cyst was performed at the same time, and three cases of retrocolonic appendix head were located under the liver. Postoperative pathology confirmed appendicitis. For patients with right upper abdominal pain and tenderness, the possibility of subhepatic appendicitis should be considered before operation. Emergency abdominal CT has more advantages than ultrasound. Laparoscopy can not only make a definite diagnosis but also perform appendectomy at the same time.

## 1. Introduction

Ectopic appendicitis is one of the rare acute abdomen in emergency surgery, especially the subhepatic type, which is often misdiagnosed as cholecystitis and other diseases, and its diagnosis and treatment are difficult. From July 2018 to December 2019, the emergency surgery department of Zhejiang Provincial People's hospital treated 6 patients with acute appendicitis under the liver. All of them underwent laparoscopic exploration + laparoscopic appendectomy with satisfactory results [1, 2]. The clinical manifestations, diagnosis, and experience of emergency laparoscopic treatment are summarized as follows.

The rest of this paper is organized as follows: Section 2 discusses data and methods, followed by experimental result in Section 3.  Section 4 concludes the paper with summary and future research directions.

## 2. Data and Methods

### 2.1. General Information

There were 6 patients in this group, 5 males and 1 female, aged from 21 to 64 years (44.2 ± 17.6 years) [3]. Medical history: the time from onset to treatment was 7∼56 h, with an average of 30.6 h. Clinical manifestations: all of them showed pain in the right upper abdomen, and other symptoms included fever (4 cases), nausea and vomiting (3 cases), radiation pain in the right shoulder and back (2 cases), diarrhea (1 case), and cessation of anal exhaust and defecation (3 cases) [4, 5]. Physical examination: deep tenderness in the right upper abdomen or right middle abdomen (5 cases), percussion pain in the right liver area (1 case) [6–8]. Auxiliary examination: blood routine leukocyte >10 × 109/L in 18 cases. Ultrasound examination in our hospital or other hospitals showed liver cyst (1 case), cholecystitis (4 cases) and appendicitis (1 case) [9]. The diagnostic rate of ultrasound was only 16.7%. All 6 patients underwent plain abdominal CT scan, all of which showed acute appendicitis, and 1 case showed liver cyst.  Table 1 is data of 6 patients.  Figure 1 is appendix with liver cyst.

### 2.2. Operation Method

All 6 patients underwent endotracheal intubation, general anesthesia, laparoscopic exploration and appendectomy [10]. First, make a 1 cm incision on the upper edge of the umbilicus, enter the trocar after pneumoperitoneum, and set the intraperitoneal pressure to 10∼13 mmHg (1 mmHg = 0.133 kPa). After pneumoperitoneum, insert a 10 mm trocar from the incision [11, 12]. The patient takes the body position with head low and feet high to the left, and places a 30° mirror [13]. Explore the abdominal visceral organs, liver, gallbladder, spleen, stomach, duodenal bulb, small intestine/colon and its mesangium, omentum, pelvic cavity, uterus and accessories, look for ectopic appendix according to the preoperative CT results, and further clarify the diagnosis of ectopic appendicitis. Intraoperative findings: peritoneal and pelvic effusion in 3 cases [14]. The root of ectopic appendix was located under the liver in 2 cases, 1 case with absence of ascending colon, and 1 case with ectopic ascending colon and transverse colon; In 4 cases, the root of appendix was located in the right lower abdomen, and the head end was located under the liver, including 1 case in the liver cyst and 3 cases in the posterior position of colon; The length of appendix is 5∼13 cm and the diameter is 1.0∼1.5 cm [15]. Two more incisions were taken according to the position of ectopic appendix, and 10 mm and 5 mm trocar were inserted respectively. One was located under the xiphoid process with 2 transverse fingers and 10 mm trocar was inserted; In the other position, take the upper and lower parts of the flat umbilicus at the front line of the right axilla and place 5 mm trocar [16]. Treatment of appendix mesangium: free the appendix, expose the whole process, treat the appendix mesangium by times, and disconnect the mesangium to the root after ligating the mesangium with vascular clamp. Treatment of appendix root: after handling the appendix mesangium, lift the appendix, double clamp the appendix with a vascular clamp at 0.5 cm away from the cecum, clamp the appendix with a vascular clamp at 1 cm away from the cecum, and cut off the appendix between them. The mucosa of the appendix stump was burned by electrocoagulation [17]. Laparoscopic fenestration and drainage of hepatic cyst was performed in 1 case.  Figure 2 is appendicitis with absence of ascending colon [18].  Figure 3 is appendicitis with ectopic ascending and transverse colon.  Figure 4 is appendix in the posterior position of colon.  Figure 5 is appendix in the posterior position of colon.  Figure 6 is appendix in the posterior position of colon.

Figure 7 is results of appendix mucosa.  Figure 8 is the observation hole shall be set between the two operation holes as far as possible.  Figure 9 is puncture hole under xiphoid process and right puncture hole.

### 2.3. Statistical Analysis

The measurement data are expressed in mean ± standard deviation, and the counting data are expressed in frequency. The data were statistically processed by SPSS 17.0 statistical software. All counting data were tested by chi square test, and the measurement data were measured by mean ± standard deviation (−*x*) ± *s*) indicates that paired *t*-test is used for intra group comparison and group *t*-test is used for inter group comparison. Inspection level *α* = 0.05, with *P* < 0.05 as the difference, the difference was statistically significant.

## 3. Experimental Result

All 6 patients in this group successfully completed laparoscopic surgery without conversion to laparotomy. The operation time was 35∼90 min, with an average of 57.5 min. The intraoperative bleeding was 5∼20 ml, with an average of 10.8 ml. abdominal drainage tubes were placed in 3 cases. The postoperative anal exhaust time was 5∼19 h, with an average of 13 h, 6∼14 h, with an average of 9.5 h. The postoperative hospital stay was 3∼5 d, with an average of 4.3 D. Postoperative pathology confirmed that there were 3 cases of acute simple appendicitis and 3 cases of suppurative appendicitis as shown in Figure 7. No abdominal and incision infection occurred after operation. The patients were followed up for 12∼20 months, with an average of 14.7 months. There were no long-term complications such as incision hernia, intestinal obstruction, abdominal and pelvic abscess, appendicitis, and fecal fistula. The therapeutic effect was satisfactory.

Ectopic appendix can be seen in the posterior position of cecum, high position, pelvic position, intramural appendix, left appendix, misplaced appendix, intracavitary appendix and hernia appendix. The incidence of subhepatic appendix is low. Palanivelu et al. Counted 7210 cases of appendicitis in India, the incidence of subhepatic appendix is 0.08%.

Most patients with appendicitis have metastatic persistent abdominal pain, and some patients show pain at the lesion site from the onset. However, due to the change and variation of anatomical position, ectopic appendix can show pain and signs in the corresponding part, and it is easy to be confused with the lesions of tissues and organs in this part. Due to the particularity of the location of the appendix, the clinical manifestation of subhepatic ectopic appendicitis is similar to hepatobiliary or gastrointestinal related diseases, mainly manifested as fixed tenderness in the liver area of the right upper abdomen colon. At the same time, inflammation can stimulate the phrenic nerve, resulting in radiation pain, Hiccup and vomiting in the right shoulder and back. Abdominal ultrasonography may cause unclear diagnosis or misdiagnosis as acute cholecystitis due to the influence of subhepatic effusion or gas in colon and duodenum caused by high position of appendix. Although ultrasound is often used for the examination of acute appendicitis, CT is more sensitive than ultrasound. Ultrasound examination in our hospital or other hospitals showed liver cyst (1 case), cholecystitis (4 cases) and appendicitis (1 case). The diagnostic rate of ultrasound was only 16.7%. CT is more useful in the diagnosis of atypical right upper abdominal pain and nonspecific clinical symptoms. All 6 cases in this group underwent abdominal CT plain scan, which all suggested appendicitis. Therefore, we believe that for patients with right upper abdominal pain and tenderness who cannot rule out ectopic appendicitis, it should be further clarified by plain CT scan before operation.

Once acute appendicitis is diagnosed, surgery should be performed as soon as possible. Laparoscopy has certain advantages in intraoperative diagnosis and treatment of acute abdomen, including clarifying the etiology of acute abdomen and the location of lesions in the abdominal cavity. It can well complete abdominal exploration and deal with abdominal adhesion and exudation. In recent years, laparoscopic appendectomy has been considered as the standard method for the treatment of acute appendicitis. The position of puncture hole is the key in laparoscopic surgery for ectopic appendicitis. Adjust the position of lens hole and operation hole according to the position of appendix root and head end. Generally, the position of the left and right operation holes follows the isosceles triangle principle. The closer the intersection angle between the left and right hand instruments is to 60°, the more in line with the ergonomic principle. The observation hole shall be set between the two operation holes as far as possible, and the distance between the observation hole and the operation hole should be more than 6 cm to avoid the collision between the lens and the operation equipment, as shown in Figure 8. For the subhepatic appendix, refer to the puncture hole during laparoscopic cholecystectomy: place the laparoscopic lens above the umbilicus, and place the 10 mm trocar under the 2 transverse fingers of the xiphoid process; In the other position, take the upper and lower parts of the flat umbilicus at the front line of the right axilla, place 5 mm trocar and place the operation hole, as shown in Figure 9. Be careful during operation to avoid damage to the liver.

## 4. Conclusion

In conclusion, for patients with right upper abdominal pain and tenderness, the possibility of subhepatic appendicitis should be considered before operation. Emergency abdominal CT has more advantages than ultrasound. Laparoscopy can not only make a definite diagnosis, but also perform appendectomy at the same time. Good puncture hole position can greatly reduce the difficulty of operation.

## Figures and Tables

**Figure 1:** Appendix with liver cyst.

**Figure 2:** Appendicitis with absence of ascending colon.

**Figure 3:** Appendicitis with ectopic ascending and transverse colon.

**Figure 4:** Appendix in the posterior position of colon.

**Figure 5:** Appendix in the posterior position of the colon.

**Figure 6:** Appendix in the posterior position of the colon.

**Figure 7:** Results of appendix mucosa.

**Figure 8:** The observation hole shall be set between the two operation holes as far as possible, and the distance between the observation hole and the operation hole shall be more than 6 cm to avoid the collision between the lens and the operation equipment.

**Figure 9:** Puncture hole under xiphoid process and right puncture hole.

**Table 1:** Data of 6 patients.

Case	Gender	Age (years)	Onset of operation time (hours)	Operation time (minutes)	Postoperative drainage time (days)	Postoperative hospital stay (days)	Intraoperative bleeding (ML)	Postoperative exhaust time (hours)	Postoperative time (day)	Postoperative follow-up time (months)
1	Male	30	12	35	2	5	5	5	6	14
2	Male	57	35	75	3	5	10	10	8	18
3	Male	21	7	40	0	4	10	15	6	20
4	Male	63	56	90	3	4	20	14	10	12
5	Male	64	32	45	0	5	10	15	14	12
6	Female	30	42	60	0	3	10	19	13	12

## Data Availability

The simulation experiment data used to support the findings of this study are available from the corresponding author upon request.
